The article "Design and Application of Sports-Oriented Public Health Big Data Analysis Platform" was published in 2022. Journal: J Environ Public Health.

# Design and Application of Sports-Oriented Public Health Big Data Analysis Platform

**DOI:** 10.1155/2022/7684320

**Published:** 2022-09-24

**Authors:** MingJun Liu, LingGang Meng, QinEr Xu, MingHua Wu

**Affiliations:** School of Physical Education, Changzhou University, Changzhou Jiangsu 213164, China

## Abstract

People's pursuit of public health continues to improve with the rapid economic development. Physical activity is an important way to achieve public health. Excessive physical activity intensity and uncomfortable forms of physical activity can affect people's physical and mental health. Reasonable physical activity intensity and reasonable physical activity form will be beneficial to public health. People need to choose the corresponding sports mode according to physical function parameters and mental health parameters. However, it is difficult to understand the relationship between physical activity patterns and public health-related parameters, which limits people to establish reasonable exercise patterns. This research uses big data technology to design an intelligent sports-oriented public health data analysis scheme. It mainly uses MLCNN method and LSTM method to extract physical function parameter features, mental health parameter features, and sports parameter features. The research results show that the MLCNN method and LSTM can accurately extract and predict the parametric features related to sports and public health. The largest relative mean error is only 2.52%, which is the predicted value of the physical performance parameter characteristics. The smallest prediction error is also 2.27%, and this part of the relative error comes from the prediction of sports parameters.

## 1. Introduction

The improvement of economic level has brought people a higher quality of life and happiness. In the era of sufficient material life, people also began to pay more attention to their health [1, 2]. People often use sports to achieve fitness goals. Public health has become a trend in today's society, which is why people continue to pay attention to physical and mental health. There are also many forms of physical exercise, and different groups of people will have different suitable sports [3, 4]. Appropriate physical activity will promote physical health, but excessive or inappropriate forms of physical activity are not only harmful to physical health; it may also cause loss of physical function [5, 6]. Therefore, reasonable sports forms and reasonable sports methods can improve people's pursuit of health. This requires people to pay more attention to the relationship between physical function and physical health, so that it can find suitable forms of sports and methods of sports [7, 8]. For young people, intense physical activity may promote the body's metabolism, which will also cultivate a positive and optimistic attitude in young people. Long-term nonparticipation in sports can easily lead to the decline of physical function and unhealthy mental state. For the elderly, appropriate physical activity will promote physical health, and it will make the elderly maintain a better mental attitude and physical function [9, 10]. However, excessive physical exercise and intense physical activity are not good for the body of the elderly. This requires the elderly to choose appropriate sports according to their physical indicators [11, 12], so as to achieve the goal of pursuing physical health. It can be seen that different groups have different requirements for sports and the intensity of sports.

The article "Design and Application of Sports-Oriented Public Health Big Data Analysis Platform" was published in 2022. Journal: J Environ Public Health.

Different groups choose appropriate sports and exercise intensity, which requires people to understand the relevant indicators of physical function and the relationship between sports and the body [13, 14]. It is difficult to understand the quantitative relationship between physical activity intensity and physical performance. Despite the rapid development of the Internet with technology and high technology, data on the relationship between physical function and physical activity are relatively scarce [12, 15]. If people can choose the relevant physical activity according to the characteristics of the body's heart rate, pulse, and fitness level, it will achieve the purpose of physical health [16, 17]. When people have a healthy body and a healthy mind, they will not only have more expectations and enthusiasm for life but also create higher goals in life. Public health mainly includes physical health and mental health. Big data technology can better establish the mapping relationship between research objects for different characteristics [18, 19]. Therefore, it is a new direction for big data technology to solve the relationship between physical exercise and physical function, mental health, and other aspects. There is a complex relationship between sports and public health-related parameters, which is a nonlinear relationship that cannot be solved by artificial means through experiments or formula methods. Big data technology can efficiently extract the characteristics between sports and public health and establish a quantitative relationship between the two.

Big data technology has shown powerful advantages in dealing with huge amounts of data, it will extract the characteristics of huge amounts of data, and it can establish connections between data [20, 21]. If big data technology is applied to sports-oriented public health, it will extract physical function indicators and characteristics of mental health, and it will also establish the relationship between physical and mental health and physical activity intensity and physical activity form [22, 23]. Big data technology can solve some problems that traditional manual methods and empirical methods cannot solve [24, 25]. It is difficult for people to deal with huge amounts of data, and there is also a relatively complex nonlinear relationship between big data, which requires big data technology to use the distribution of weights and biases to establish nonlinear relationships between research objects. In life and production, there are often complex nonlinear relationships between the characteristics of research objects. These relationships are difficult to establish through empirical formulas, and big data technology is used for processing and prediction [26, 27]. So far, big data technology has more mature algorithms for feature extraction and feature prediction [28, 29]. This provides more convenience for the application of big data technology in various life and production fields.

The article "Design and Application of Sports-Oriented Public Health Big Data Analysis Platform" was published in 2022. Journal: J Environ Public Health.

This study uses big data technology to establish the relationship between sports characteristics and physical and mental health characteristics, and it also designs an intelligent public health big data platform. This study mainly designs a multipath convolutional neural network (MPCNN) and LSTM neural network to extract features related to public health and sports. First, this study introduces the relationship between physical activity and physical and mental health in Section 1; it also introduces the relevant research background of big data technology.  Section 2 describes the current state of research in public health and sports. The platform for the relationship between intelligent physical activity and physical and mental health designed in this study using MPCNN and LSTM is introduced in Section 3.  Section 4 highlights the reliability of MPCNN and LSTM methods in predicting and extracting features related to sports and public health. This study summarizes and analyzes the application value and reliability of big data technology in sports-oriented public health platform in Section 5.

## 2. Related Work

Although physical exercise can promote the development of physical and mental health, it puts forward requirements for the intensity of physical exercise and the way of physical exercise. Different groups of people are suitable for different sports intensities and different forms of sports. This requires the selection of relevant sports forms according to one's own physical function and mental state. Many researchers have studied the relationship between physical activity and public health. Yuan [30] has found that physical activity improves fitness and also improves mental health in college students. However, it was also found that the current college sports facilities that are not complete can hinder the development of college students' physical and mental health through sports. This study uses literature survey method, Delphi method, and factor analysis method to study the relationship between physical and mental health and physical activity of college students. The results of the study found that factors such as study pressure and family will affect the physical and mental health of students, which requires reasonable physical exercise to improve physical and mental health. Liu et al. [31] mainly explore the relationship between urban public settings and public health. The shortage of urban public sports facilities has limited the healthy development of public sports. However, little research has been conducted to comprehensively assess the relationship between urban physical activity and public health. This study uses multisource urban data and GIS network analysis method to quantitatively analyze the relationship between urban sports and public health. The results of the study found that reasonable urban sports facilities will also promote the development of public health, which will promote people's pursuit of physical and mental health. The multisource data model proposed in this study also has certain value for studying public health. Schneider et al. [32] mainly analyze climate change and the relationship between physical activity and public health. They mainly explore the impact of extreme weather, ultraviolet rays, allergens, and other factors on public physical and mental health. They use the sport, club, and climate change model (SC3 model) to develop a conceptual model to study the relationship between climate change and physical and mental health risks. These public health assessments mainly include early warning systems and coordinated assessment systems. The results show that the SC3 model can predict the risk relationship between climate change and physical and mental health, which has an important role for people to improve physical and mental health and reduce the impact of climate on physical and mental health. Liu and Zhang [33] also believe that reasonable sports facilities will improve people's well-being; it will also improve people's physical and mental health. However, the layout of sports facilities is unreasonable and the gap between urban and rural areas is large. This study uses big data technology and visual methods to study the layout of urban public health-related sports facilities. This approach primarily quantifies issues such as diversity and coordination in sports settings. The research results show that the space utilization rate of sports facilities designed by this big data method is improved by 15.32%. This method can maximize the utilization rate of the city, and it can also improve people's pursuit of health. Baghapour et al. [34] study mainly analyzed the relationship between swimming and public health. This study uses the multicriteria decision-making method and fuzzy OWA method in big data technology to analyze the relationship between the environment and health of swimming pool construction. Swimming is also a form of physical activity that improves health. The results of the study found that the expansion index would be useful for studying the qualitative relationship between swimming exercise and health. From the above review, it can be seen that few researchers use big data technology to analyze the characteristics of public health or sports. This study will use big data technology to quantitatively analyze the correlation between sports and public health.

The article "Design and Application of Sports-Oriented Public Health Big Data Analysis Platform" was published in 2022. Journal: J Environ Public Health.

## 3. Analysis and Application of Big Data Technology in Sports-Oriented Public Health Platform

### 3.1. The Importance of Big Data Technology for Public Health Analysis

There is a strong correlation between physical function parameters and mental health and the intensity of physical activity and the way of physical activity. However, it is difficult for people to quantitatively analyze the relationship between physical function parameters and sports characteristics, which limits people's pursuit of public health. This study uses MLCNN and LSTM methods to build an intelligent sports-oriented public health data analysis platform. The MLCNN method can extract features such as physical function parameters and mental health indicators related to public health, which can establish a nonlinear relationship between public health-related features and sports features. LSTM methods can extract temporal features related to public health. The MLCNN method and the LSTM method can jointly extract the spatial and temporal features related to public health. Most traditional methods have difficulty considering the relationship between public health-related characteristics and time. The hybrid MLCNN-LSTM method can comprehensively consider various nonlinear relationships of features. This allows for a more precise understanding of the relationship between public health characteristics and sports parameters.

### 3.2. Application of MLCNN Algorithm and LSTM Algorithm in Sports-Oriented Public Health Data Analysis

This research intends to use MLCNN method and LSTM algorithm to realize the intelligent analysis platform of sports and public health-related parameters. If this kind of intelligent public health data analysis platform is established and trained, people can carry out relevant sports activities according to their physical function parameters and mental health indicators. This can better guide people to pursue physical and mental health. This study mainly studies three characteristics of public health physical function parameters, mental health indicators, and sports parameters. In this study, a large number of datasets collected will be classified according to different weights.  Figure 1 shows the workflow of the MLCNN method and the LSTM algorithm in extracting and predicting features related to public health and sports parameters. First, this intelligent platform divides the vast datasets it collects into three broad categories. These three types of data represent the characteristics of physical function parameters, the characteristics of mental health indicators, and the characteristics of sports parameters. After the data of these three features is processed, it will be input to the input layer of MLCNN for feature extraction process. The MLCNN method will contain multiple input layers, which can extract public health-related features at different scales. Then, these extracted features are again input to the input layer of LSTM for the extraction process of common health time-related features. For the MLCNN-LSTM algorithm, convolution operations and an iterative process are required in the training phase. However, the convolution operation is not performed in the test phase; it is only a matrix operation with weights and biases.

The article "Design and Application of Sports-Oriented Public Health Big Data Analysis Platform" was published in 2022. Journal: J Environ Public Health.

### 3.3. Basic Principles and Network Design of MLCNN and LSTM Algorithm

The working principle of MLCNN method and CNN method is similar. CNN methods utilize convolutional layers, pooling layers, and activation functions for feature extraction and transformation of nonlinear relationships. The MLCNN algorithm consists of three paths. It mainly consists of two paths that do not contain pooling layers. It only contains convolutional layers. The other path consists of pooling layers and convolutional layers. The pooling layer designed in this study adopts the method of maximum pooling layer. Compared with the single-path CNNF method, the MLCNN method can extract more features, and it can also extract features of different scales. This is beneficial to the data analysis of sports-oriented public health platforms, because the data related to public health is relatively complex.  Figure 2 shows the working path of the MLCNN method. The pooling layer can reduce the operation parameters of the deep learning framework, and it can also extract relevant features from different angles and paths. It can be seen from Figure 2 that the MLCNN algorithm contains three paths, which include two single CNN algorithm paths and a neural network path with a maximum pooling layer. The three paths will be concatenated through a fully connected layer. In this study, the MLCNN method is similar to the CNN method and it also contains more parameters. The number of filters, sliding step size, and learning rate of the MLCNN method designed in this study are 256, 1, and 0.0001, respectively.

The article "Design and Application of Sports-Oriented Public Health Big Data Analysis Platform" was published in 2022. Journal: J Environ Public Health.

A sports-oriented public health data analysis platform will also involve time-related features. If the temporal features of public health-related features are not extracted, this will ignore the data analysis of time for public health. The LSTM method can memorize some historical information data, but it does not memorize all temporal features. If the LSTM algorithm memorizes the state data at all times, it will cause the data complexity and reduce the training speed of the deep learning framework. The LSTM algorithm can selectively filter and select the information data at all times, and it will leave the historical data with greater influence according to the distribution of weights. This is due to the specific gate structure of LSTM.  Figure 3 shows the working scheme of the LSTM method for selecting information. It can be seen from Figure 3 that the output layer of the LSTM method is connected to the forgetting layer and the input layer of the next LSTM layer. The LSTM algorithm contains three neural network layers.

### 3.4. Mathematical Theory and Mathematical Principles of MLCNN Algorithm and LSTM Algorithm

This study uses the MLCNN-LSTM algorithm to extract the features related to sports and public health, which mainly involve physical function parameter features, mental health parameter features, and sports parameter features. The MLCNN method can be extracted from multiple angles and dimensions and public health-related characteristics. The detailed calculation process is as follows.

Both MLCNN and CNN methods involve convolution operations in both intelligent algorithms. The convolution operation will calculate the relationship between the data of the input feature and the convolution operator. Expression (1) and Expression (2) show the two steps of the convolution operation process. Expression (1) computes the integral operation of convolution. Expression (2) shows the sum operation of the convolution operation. Expression (3) shows the overall calculation process of the convolution operation.

(1) $$\begin{array}{c} \int_{-\infty }^{\infty }f\left(\tau \right)g\left(x-\tau \right)d\tau , \end{array}$$

(2) $$\begin{array}{c} \int_{0}^{\tau }f\left(x\right)g\left(\tau -x\right)dx, \end{array}$$

(3) $$\begin{array}{c} \left(f*g\right)\left(x\right)=\int_{-\infty }^{\infty }f\left(t\right)g\left(x-t\right)dt. \end{array}$$

Expression (4) shows the convolution calculation process of MLCNN, which also reflects the calculation process between weights and biases and parameters. Expression (5) shows the derivation process of MLCNN. Weights are related operations according to the gradient descent method, and derivation is a basis of gradient descent.

(4) $$\begin{array}{c} x_{j}^{\ell }=f\left(\underset{i\in M}{\sum }x_{i}^{\ell -1}*k_{ij}^{\ell }+b_{j}^{\ell }\right), \end{array}$$

(5) $$\begin{array}{c} \frac{\partial J}{\partial b_{j}^{l}}=\underset{uv}{\sum }\left(\delta_{j}^{l}\right)=\frac{\partial J}{\partial z_{j}^{l}}*\frac{\partial z_{j}^{l}}{\partial b_{j}^{l}}. \end{array}$$

Expression (6) shows the derivation process of the bias. The distribution of bias and weight is a manifestation of the nonlinear relationship, which is also a basic algorithm of gradient descent. Expression (7) shows the calculation rule of the size of the output feature, which mainly involves parameters such as filter and sliding step size.

(6) $$\begin{array}{c} \frac{\partial E}{\partial k_{ij}^{l}}=\underset{uv}{\sum }\left(\delta_{j}^{l}\right){\left(P_{I}^{\ell -1}\right)}_{uv}, \end{array}$$

(7) $$\begin{array}{c} w^{\prime }=\frac{\left(w+2p-k\right)}{s}+1. \end{array}$$

The optimal weight distribution and optimal bias distribution are done using the gradient descent method. The gradient descent method will iterate to find the region of the global minimum. Expression (8) shows the calculation rules of the gradient descent method. Whether it is MLCNN or LSTM algorithm, it will involve the gradient descent method.

(8) $$\begin{array}{c} d_{j}^{\ell }=\text{down}\left(x_{j}^{\ell -1}\right). \end{array}$$

Expression (9) shows the calculation method of the forget gate of the LSTM neural network. The forget gate will select and filter the historical information according to the size of the weight and the influence on the current state information.

(9) $$\begin{array}{c} f_{t}=\sigma \left(w_{f}\cdot \left[h_{t-1},P_{t}\right]+b_{f}\right). \end{array}$$

Expression (10) shows the calculation rule of the input gate of the LSTM algorithm. The input gate will control the input of historical information and current information, and the information will be used as new input data through the input gate. Expression (11) and Expression (12) show the update gate and output gate rules of the LSTM algorithm. The update gate is responsible for updating the values of the weights. The output gate complex selectively feeds data into the next layer of the neural network.

(10) $$\begin{array}{c} i_{t}=\sigma \left(\omega_{i}\cdot \left[h_{i-1},P_{t}\right]+b_{i}\right), \end{array}$$

(11) $$\begin{array}{c} {\overset{⟶}{C}}_{t}=f_{t}\times {\overset{⟶}{C}}_{t-1}+i_{t}\times {\overset{⟶}{C}}_{t}, \end{array}$$

(12) $$\begin{array}{c} O_{t}=\sigma \left(w_{o}\cdot \left[{\overset{⟶}{h}}_{t-1},P_{t}\right]+b_{o}\right). \end{array}$$

The article "Design and Application of Sports-Oriented Public Health Big Data Analysis Platform" was published in 2022. Journal: J Environ Public Health.

## 4. Result Analysis and Discussion

This study uses big data technology to build a special data analysis platform related to sports and public health, which is a method for quantitative data analysis. The task of feature extraction with big data technology requires a large amount of data as data support, and a large amount of data is also the basis for big data technology to learn data correlation. MLCNN and LSTM methods can find and build nonlinear relationships from a large amount of sports and public health-related data. At the same time, the more feature types the dataset contains, the more knowledge about sports and public health can be learned by big data technology. If the dataset is too small, this will not only reduce the generalization ability of MLCNN and LSTM algorithms in sports and public health applications but also easily cause overfitting. If the number of datasets is too large, this will result in wasted data and increased training time. This study selected the data related to sports and public health in Beijing. Beijing's sports and public health data will contain more features than other provinces, because Beijing's medical level and urban facilities are more developed. Datasets about people are also easy to collect.

Both the CNN method and the MLCNN method can complete the feature extraction of parameters related to sports and public health. CNN and MLCNN methods have different performances on different datasets. This study first compares the performance of CNN-LSTM and MLCNN-LSTM methods in extracting sports and public health-related parameters. First, this study analyzes the performance of two big data techniques in public health forecasting using a global measure of mean relative error.  Figure 4 shows the average relative error of the CNN-LSTM algorithm in predicting three parametric features of sports and public health. It can be seen from Figure 4 that the CNN-LSTM method can also accurately extract the characteristics of physical function parameters, mental health characteristics, and sports parameters. The prediction errors of the three different characteristics are all within 3%. The error has already met the error range of people's prediction of sports and public health-related characteristics. The prediction error of the physical function parameter feature is only 2.89%, which is the largest part of the feature. The relationship between physical function and physical activity was more complex than the other two health characteristics, which led to larger prediction errors. The prediction error for features related to mental health parameters was only 2.55%. Through the above analysis, it can be found that the CNN-LSTM method can analyze the relevant data of public health.

The article "Design and Application of Sports-Oriented Public Health Big Data Analysis Platform" was published in 2022. Journal: J Environ Public Health.

This study also compares the differences between the CNN-LSTM method and the MLCNN-LSTM method in extracting and predicting sports and public health-related features.  Figure 5 shows the average relative error distributions for the three characteristics of sports and public health. In Figure 5, every two histograms represent a feature related to sports and public health; from left to right are physical function parameter features, mental health parameter features, and sports parameter features. The left side represents the relative mean prediction error using the CNN-LSTM method. It can be clearly seen from Figure 5 that the error range of the three characteristic parameters of sports and public health has been reduced. For the features of physical function parameters, the average relative error was reduced from 2.89% to 2.52%, and this part of the error was reduced by 0.37%. This relative percentage was relatively large despite the low level of reduction in the physical performance parameter characteristics. The magnitude of the reduction in this part of the error is extremely beneficial to the discovery of physical function and the intensity and type of physical activity. For the mental health parameter features, the average relative error of this part was reduced from 2.55% to 2.27%. This part of the error reduction range is 0.28%. The average relative error of sports parameter features was reduced from 2.72% to 2.47%. It can be found through the above research that the MLCNN-LSTM method is more suitable for data analysis of sports and public health. The MLCNN method can extract relevant features of public health and sports from multiple perspectives and multiple paths. CNN methods only extract public health features from one path, which leads to large prediction errors.

From the Figures 4 and 5, it can be confirmed that the MLCNN-LSTM method used in this study has higher accuracy. The relative mean error is correlated from the perspective of global prediction accuracy, and this study also analyzes the local prediction accuracy of each feature individually. First, this study selected 35 groups of different physical function parameters for error analysis.  Figure 6 shows the prediction error distribution of the physical function parameter features. In Figure 6, the abscissa represents a straight line with a prediction error of 2%. The upper part of the abscissa represents that the prediction error of physical function parameters is more than 2%. The lower part of the abscissa represents that the prediction error of physical function parameter characteristics is less than 2%. It can be seen from Figure 6 that the characteristics of 35 different groups of physical function parameters are all distributed below 3%. Half of the physical function parameter features are distributed below 2%. Only one in seven data points had a forecast error of more than 3.5%, but the distribution of these data points was also within a reasonable margin of error. It can be seen from Figure 6 that the prediction error range of physical function parameter features is between 0 and 3.5%. The reason for the large error range in this part may be that the dataset of physical function parameters has relatively large fluctuations. Overall, the MLCNN-LSTM method can also accurately predict different physical function parameters. Not only does it have superior performance in global body function parameter features; it also has high accuracy for each body function parameter indicator. This can be very helpful to people to discover the relationship between bodily function and public health.

The article "Design and Application of Sports-Oriented Public Health Big Data Analysis Platform" was published in 2022. Journal: J Environ Public Health.

This study also selected 35 different groups of mental health parameters for local predictive analysis. Mental health parameters vary greatly. For different groups of people, mental health status also affects the intensity and type of physical activity. Physical activity can promote the development of mental health. Therefore, it is also an advantageous way for people to understand the relationship between mental health parameters and physical exercise parameters.  Figure 7 shows the change trend of the prediction curve of mental health parameter characteristics. In Figure 7, the blue curve represents the predicted value distribution of the mental health parameter feature, and the yellow curve represents the actual value distribution of the mental health parameter feature. It is used to verify the performance and reliability of the MLCNN-LSTM method. It can be seen from Figure 7 that the data of the mental health parameter characteristics fluctuates greatly. However, the predicted values of the mental health parameter characteristics are in good agreement with the actual data values. The MLCNN-LSTM method can not only predict the value of the parameters of mental health, but it can also predict the trend of the parameters of mental health. Whether it is the peaks and troughs of mental health parameters, this intelligent algorithm can accurately predict. It can be seen from the above analysis and research that this method can also help people to establish the relationship between mental health parameters and physical activity.

The article "Design and Application of Sports-Oriented Public Health Big Data Analysis Platform" was published in 2022. Journal: J Environ Public Health.

The data analysis of sports and public health involved in this study mainly includes three characteristics: physical function parameters, mental health parameters, and sports parameters. Similarly, this study also selected 35 sets of data for local predictive analysis of sports parameters. If the MLCNN-LSTM algorithm can accurately predict the characteristics of sports parameters, it can successfully help different groups to choose appropriate sports forms and sports intensity, which can really help people to achieve the goal of pursuing public health.  Figure 8 shows the prediction of sports parameter features for 35 different groups of population data. It can be seen from Figure 8 that the MLCNN-LSTM algorithm has high accuracy in predicting 35 different sets of sports parameters. Similar to the characteristics of mental health parameters, the characteristics of sports parameters also have relatively large fluctuations, and there are many peaks and troughs. It can be seen from Figure 8 that the characteristic data of sports parameters has a small prediction error at the trough, but there is a relatively large prediction error at the peak of the sports characteristic data. However, this part of the error is also acceptable for public health research. Although the trend of peaks and troughs is detrimental to the performance of MLCNN-LSTM, it can improve the generalization ability of this intelligent algorithm. The reason for the large difference between the peaks and troughs of sports-related parameters may be the large gap between the eigenvalues of the sports intensity and the sports form, which will lead to a large difference in the weight distribution in the data processing stage. Overall, the MLCNN-LSTM method can meet people's needs for data analysis of sports parameters.

## 5. Conclusions

With the continuous improvement of the quality of life, people begin to pursue physical health. They also realize the importance of physical and mental health for life and productive activities. Physical activity is an important way to improve physical and mental health. However, excessive physical activity intensity or uncomfortable forms of physical activity are detrimental to public health. Only when people choose the appropriate form of physical activity according to their physical function parameters and mental health parameters can they be beneficial to the realization of public health purposes. However, it is difficult to understand the relationship between public health parameters and sports parameters, which can limit the development of public health goals. With the development of big data technology, it provides possibilities and support for sports-oriented public health data analysis. The parameters involved in sports and public health are relatively complex, and the amount of data on the characteristics of this research object is also relatively large. Big data technology can successfully process the data and features contained in sports parameters.

The article "Design and Application of Sports-Oriented Public Health Big Data Analysis Platform" was published in 2022. Journal: J Environ Public Health.

This research uses the MLCNN algorithm and LSTM algorithm in big data technology to design an intelligent sports and public health data analysis scheme. These two algorithms can fully extract the features of physical function parameters, mental health parameters, and sports parameters, and it can also help people establish the relationship between sports and public health. First, this study compares the differences between the CNN-LSTM algorithm and the MLCNN-LSTM algorithm in predicting public health and sports characteristics. Through research, it can be found that the MLCNN-LSTM algorithm has higher accuracy than the CNN-LSTM algorithm. For the features of physical function parameters, the average relative error was reduced from 2.89% to 2.52%. For the mental health parameter feature, the mean relative error was reduced from 2.55% to 2.27%. The prediction error of sports parameter features has also been greatly reduced. The characteristics of physical function parameters and mental health parameters are two important characteristics related to public health. The prediction error of physical function parameter features is reduced by 0.37%. Compared with the CNN-LSTM algorithm, the prediction error of mental health parameter features is reduced by 0.28%. In general, the MLCNN-LSTM method is suitable for building a sports-oriented public health data analysis platform. The sports-oriented public health data analysis platform designed in this study can maintain stability and reliability once it is trained. People can understand the appropriate form and intensity of physical activity according to their own body index parameters. This has relatively high practical value.

## Figures and Tables

**Figure 1:** Application of MLCNN algorithm and LSTM algorithm in extracting spatiotemporal features of public health.

**Figure 2:** Design path and working principle of the MLCNN method.

**Figure 3:** Working scheme of the LSTM method for selecting information.

The article "Design and Application of Sports-Oriented Public Health Big Data Analysis Platform" was published in 2022. Journal: J Environ Public Health.

**Figure 4:** Prediction errors of public health and sports features using the CNN-LSTM method.

**Figure 5:** Prediction errors of public health and sports features using the MLCNN-LSTM method.

**Figure 6:** Prediction error distribution of physical function parameter features.

**Figure 7:** Predictive trends of mental health parameter characteristics.

**Figure 8:** The changing trend of sports parameter characteristics.

## Data Availability

The data used to support the findings of this study are available from the corresponding author upon request.

## References

[1] Long X., Xun L. (2019). Construction of community sports public health platform from the perspective of “Internet +” and “Healthy China”. *Shandong sports science and technology.*.

[2] Zhan K. (2020). Sports and health big data system based on 5G network and Internet of Things system. *Microprocessors and Microsystems*.

[3] Jinguo D. The theoretical construction and application system development study of sports information management.

[4] Kumar H., Manoli A. E., Hodgkinson I. R., Downward P. (2018). Sport participation: from policy, through facilities, to users’ health, well-being, and social capital. *Sport Management Review*.

[5] Tianyu G., Jiawei L. (2019). Review and outlook: commentary and research on public service of youth sports health in China. *Journal of Guangzhou Institute of Physical Education.*.

[6] Bantjes J., Swartz L. (2018). Social inclusion through para sport: a critical reflection on the current state of play. *Physical Medicine and Rehabilitation Clinics of North America*.

[7] Xiong L., Zhang L., Kong Q. (2018). Rural public sports service supply-side internal demand and path orientation of reform and governance. *China Institute of Sport Science*.

[8] Clinton-McHarg T., Gonzalez S., Milner S. (2019). Implementing health policies in Australian junior sports clubs: an RCT. *BMC Public Health*.

[9] Braksiek M., Thormann T. F., Wicker P. (2021). Intentions of environmentally friendly behavior among sports club members: an empirical test of the theory of planned behavior across genders and sports. *Frontiers in Sports and Active Living*.

[10] Khan A., Hussain J., Bano S., Chenggang Y. (2020). The repercussions of foreign direct investment, renewable energy and health expenditure on environmental decay? An econometric analysis of B&RI countries. *Journal of Environmental Planning and Management*.

[11] McCullough B., Orr M., Watanabe N. M. (2020). Measuring externalities: the imperative next step to sustainability assessment in sport. *Journal of Sport Management*.

[12] Guo X., Hu A., Jian D., Chen D., Zou W., Wang Y. (2018). Urban-rural disparity in the satisfaction with public sports services: survey-based evidence in China. *The Social Science Journal*.

The article "Design and Application of Sports-Oriented Public Health Big Data Analysis Platform" was published in 2022. Journal: J Environ Public Health.

[13] Watts N., Amann M., Arnell N. (2021). The 2020 report of The _Lancet_ Countdown on health and climate change: responding to converging crises. *Lancet*.

[14] Salarvandian F., Hosseini S. A., Moradi A., Karoubi M. (2020). Assessing the spatial distribution of sports spaces within walking distance in Tehran. *International Journal of Urban Sciences*.

[15] Ibsen B., Levinsen K. (2019). Collaboration between sports clubs and public institutions. *European Journal for Sport and Society*.

[16] Zhou L., Wang J. J., Chen X., Cianfrone B., Pifer N. D. (2020). Communitysport service provision, participant satisfaction, and participation experience and perspective of Guangdong, China. *International Journal of Sports Marketing and Sponsorship*.

[17] Seidel G., Meyer A., Lander J., Dierks M. L. (2020). Facetten von Gesundheitskompetenz. *Pravention Und Gesundheitsforderung*.

[18] Evans A., Barker-Ruchti N., Blackwell J. (2021). Qualitative research in sports studies: challenges, possibilities and the current state of play. *European Journal for Sport and Society*.

[19] Jones N., Byrne L., Carr S. (2020). If not now, when? COVID-19, lived experience, and a moment for real change. *The Lancet Psychiatry*.

[20] Qiu C., Huang Q., Pan G., He X. (2022). Framework for a variational Bayesian convolutional network for velocity field prediction and uncertainty quantification of a pump-jet propulsor. *Physics of Fluids*.

[21] Zhao Y. T., Zhang Z., Feng T. W., Tao K. T. (2019). Big data development, institutional environment, and government governance efficiency. Manage. *World*.

[22] Zheng L. Y., Zhou H. W. (2019). Firm’s big data capability: a literature review and prospects. *Journal of Science and Technology Policy Managemen*.

[23] Zou Y., He W., Zhang L., Ni J., Chen Q. (2019). Research on privacy protection of large-scale network data aggregation process. *International Journal of Wireless Information Networks*.

[24] Aceto G., Persico V., Pescapé A. (2020). Industry 4.0 and health: Internet of Things, big data, and cloud computing for healthcare 4. *Journal of Industrial Information Integration*.

[25] Agarwal M., Srivastava G. M. S. (2019). “Big” data management in cloud computing environment. *Harmony search and nature inspired optimization algorithms*.

[26] Chaudhary R., Aujla G. S., Kumar N., Rodrigues J. J. P. C. (2018). Optimized big data management across multi-cloud data centers: software-defined-network-based analysis. *IEEE Communications Magazine*.

[27] Dehghani M., Ghiasi M., Niknam T., Kavousi-Fard A., Shasadeghi M., Ghadimi N. (2021). Blockchain-based securing of data exchange in a power transmission system considering congestion management and social welfare. *Sustainability*.

The article "Design and Application of Sports-Oriented Public Health Big Data Analysis Platform" was published in 2022. Journal: J Environ Public Health.

[28] Grander G., da Silva L. F., Santibañez Gonzalez E. D. R. (2021). Big data as a value generator in decision support systems: a literature review. *Revista de Gestão*.

[29] Gupta S., Godavarti R. (2020). IoT data management using cloud computing and big data technologies. *International Journal of Software Innovation (IJSI)*.

[30] Yuan M. (2021). Empirical analysis and intervention research on college students' health influence mechanism from the perspective of public sports. *Revista Brasileira de Medicina do Esporte*.

[31] Liu Y., Wang H., Sun C., Wu H. F. (2022). Equity measurement of public sports space in central urban areas based on residential scale data. *International Journal of Environmental Research and Public Health*.

[32] Schneider S., Winning A., Grueger F. (2022). Physical activity, climate change and health-a conceptual model for planning public health action at the organizational level. *International Journal of Environmental Research and Public Health*.

[33] Li W., Zhang W. (2021). Design model of urban leisure sports public facilities based on big data and machine vision. *Journal of Sensors*.

[34] Baghapour M., Moeini Z., Shooshtarian M. (2021). A new computer-based index for swimming pools' environmental health assessment in big data environment by consensus-based fuzzy group decision-making models. *Journal of Environmental Health Science and Engineering*.

